# Impact of the digital economy on urban green growth: Empirical evidence from China

**DOI:** 10.1371/journal.pone.0296072

**Published:** 2023-12-21

**Authors:** Yangjun Ren, Ze Tian, Chao Liu

**Affiliations:** 1 School of Economics and Trade, Changzhou Vocational Institute of Textile and Garment, Changzhou, China; 2 Business School, Hohai University, Nanjing, China; University of Sargodha, PAKISTAN

## Abstract

Using the digital economy to empower urban economic green growth provides essential opportunities for China to achieve high-quality growth. This paper assesses the level of digital economy and green growth in Chinese cities, seeking to explore the mechanisms and effects of the digital economy on urban green growth in a unified framework. The results indicate that the digital economy can drive cities’ green growth. This conclusion still holds after a set of robustness tests. Meanwhile, the green value of the digital economy is fully released among the eastern cities, major urban agglomerations, and high-level cities. Further research shows that the digital economy can indirectly enhance urban green growth in the neighboring regions through spatial spillover effects. Moreover, labor resource mismatch, capital resource mismatch and green technology innovation are significant mediating mechanisms. The findings could guide policymakers on green growth in emerging economies from a digital economy perspective.

## Section 1: Introduction

The booming digital economy has injected new momentum into global economic development and emerged as a key engine for global economic recovery over the past decade [1]. The digital economy scale of 47 major economies reached 38.1 trillion USD in 2021, accounting for 45.0% of GDP. The United States and the European Union have built their worldwide supremacy in the digital economy via technical innovation. Moreover, China, an emerging country, is hastening the integration of the digital economy and the real economy, building a digital industry agglomeration with international competitiveness and ranking second in the world in terms of industrial scale [2]. Unlike the traditional economy, the digital economy, with its new development pattern, is deeply integrated into all sectors of the economy and society, playing a crucial role in enhancing innovation efficiency and driving industrial transformation [3]. Furthermore, the digital economy has a unique characteristic of being environmentally friendly, and the information technology innovation it has triggered has provided the world with a useful way of exchanging information and accelerated the economic structure’s adjustment, which coincides with the prerequisites of attaining green growth [4]. Existing research indicates that green is an inherent attribute of the digital economy, such as lower marginal costs, lower resource consumption and less pollution.

Nowadays, the global economy has entered an unprecedented phase of digital transformation; it facilitates the deconstruction and reorganization of existing industrial chains, hence providing higher security, stability and efficiency than traditional chains. The exponential evolution and accessibility of digital technology have alleviated ecological pressure, providing an innovative internal development engine [5, 6]. In addition, the digital economy’s typical characteristics, such as permeability, platforming, and sharing, can optimize the industrial structure, increase resource efficiency, reduce pollution, and facilitate increased integration with low-carbon and green growth [7]. Even though the new wave of digital technology will result in a substantial digital dividend, the rising resource constraints in countries or regions worldwide imply that environmental factors should be included in the framework for evaluating economic progress. Green growth that reconciles economic progress and environmental conservation is consequently a matter of worldwide consensus [8, 9].

As the world’s largest consumer of resources, China is still in the grip of its substantial reliance on energy and the environment. Nowadays, China’s growth has entered a new phase. However, a number of issues make it difficult to sustain the rough economic development model, such as intensifying environmental pollution, tightening factor endowments, diminishing labor dividends, and declining return on capital [10, 11]. With the wide penetration of digital economy applications, the typical characteristics of regional economic development have changed dramatically; meanwhile, the digital economy has emerged as a huge potential for nations to increase their economic strength [12]. It is notable that policies concerning the digital economy and sustainable growth have been frequently incorporated into China’s critical national plans. However, the existing studies have not provided a coherent framework for answering the issue of how the digital economy drives urban green growth. This research addresses three specific questions. First, can the digital economy promote urban green growth in emerging economies? Second, if the effects are validated, what are the mechanisms behind them? Finally, what are the differences in the influence of the digital economy on cities’ green growth based on their own characteristics and spatial regions? Considering China’s pursuit of green growth and industrial modernization, it is crucial to examine the relation between the digital economy and cities’ green growth to strategically exploit the digital economy’s green value. Possible actions that can enhance the digital economy’ green effect are proposed and can serve as a guide for policymakers.

Accelerating the digital economy’s advancement contributes to energy-saving and emission-reduction, thereby improving green economic efficiency [13]. The application of digital technology can guide green technology innovation and productivity, thereby changing consumption patterns and promoting sustainable economic development [14]. Therefore, the marginal contribution of this research is threefold: firstly, this research incorporates the digital economy and urban green growth within a unified framework, providing researchers with a new perspective to investigate the limited but emerging literature. This research further investigates the mediating role of resource mismatch and green technology innovation to better understand the mechanisms by which the digital economy promotes urban green growth. Secondly, a city-level digital economy evaluation system from the four dimensions of digital industrialization, industrial digitization, digital governance, and digital sustainability is constructed to assess the digital economy level of 279 Chinese cities from 2012 to 2021. This comprehensive index contains more information and represents China’s digital economy in a multifaceted manner. Finally, a spatial econometric model is employed to thoroughly examine whether the spatial spillover effects of the digital economy on urban green growth occur. In addition, this research contributes to explore the heterogeneous impact of the digital economy on urban green growth to support the richness of our findings.

The rest of this research is arranged as follows. Section 2 reviews the relevant literature and develops our hypotheses. Section 3 details the data, variables and models. Section 4 provides the empirical findings and discussion. Section 5 concludes the paper and provides corresponding policy implications.

## Section 2: Literature review and hypotheses development

### 2.1. Literature review

The digital economy is a fresh and dynamic economic form with digital technologies at its core and computers and the Internet as its carrier. With the continuous updating and iteration of digital technologies, the digital economy has evolved into a vital driving force in reshaping the economic structure of the world [15].

Hence, research on the digital economy is also emerging, the basic concept of which was first presented by Tapscott [16], and has become increasingly inclusive and multidimensional after being widely used by academic circles. As digital infrastructure and information processing technologies continue to develop, a new generation of digital technologies such as the Internet of Things, blockchain and artificial intelligence continue to penetrate all aspects of modern economic development, and the content and connotation of the digital economy are becoming even richer and diversified [17]. Existing research implies that the core of digital technologies can empower management transformation in enterprises and help them build a competitive advantage [18]. It can also facilitate industries’ digital and intelligent upgrading and exert a powerful pull for economic growth [19]. In addition, it can strengthen digital governance [20] and improve resilience in social development. As definitions of the digital economy vary, there needs to be a consensus on how to measure it. Most studies on calculating the digital economy are qualitative [21], while its quantitative assessment can be typically divided into direct and comparative methods, which are mainly limited to the macro level, such as national and provincial [22, 23]. The measurement methods mainly include the use of the entropy value method or principal component analysis for evaluation based on the construction of an indicator system, as well as the use of efficiency analysis to indirectly reflect the regional digital economy level by estimating its output efficiency [24].

Green growth has always been a global concern, and many studies consider green economic efficiency (GEE) to be an indicator to represent regional green growth level [25, 26]. GEE can reflect the core of increasing economic quality and promote the formation of a green economic model [27]. It can also take into account ecological environment factors and unexpected outputs such as pollution emissions, which aligns with the concept of green growth in the background of times. Compared with GEE, traditional economic efficiency (TEE) cannot comprehensively measure the quality of economic growth as it does not incorporate resource and environmental factors into the productivity analysis framework [28, 29]. Given the advantages of the slack-based measure (SBM) in nonparametric methods, it has been used to assess GEE in recent years [30]. Furthermore, most of the previous literature on green growth has concentrated on different aspects of GEE, which can be impacted by environmental regulation, carbon emissions, industrial structure, digital finance, and digital economy [31–33]. Most scholars believe that technological innovation should be prioritized as the main strategies for promoting green growth [34]. However, studies have yet to investigate its influence factors from a technical standpoint. Technological innovation can considerably reduce pollution emissions, and green technology innovation is a primary goal for improving GEE.

As a technology-intensive activity, the digital economy has become profoundly ingrained into economic progress, provoking a macro-level analysis of its effects. Thus, researchers have aimed to evaluate GEE and explore what drives the digital economy. However, there is a relative lack of studies linking the digital economy to cities’ sustainable growth. Its impact and potential mechanisms can only be deduced from other relevant research. Nguyen and Su [35] found that the digital economy can apply digital technologies to upgrade the industrial structure, and promote industries’ digital development and green transformation. Pan et al. [36] claimed that the digital economy could increase the capacity for innovation and companies’ productivity and enhance the greening of economic activities. Furthermore, studies on the relation between the Internet and economic advancement can offer a reference for analyzing the effects of the digital economy on green growth. Some scholars hold that the Internet’s development can enhance regional technological innovation, improve regional resource mismatch and promote the industrial restructuring to achieve emission reduction [37, 38]. However, the Internet may have varying effects on the green growth of regions at different economic levels [39, 40]. In addition, the relation between the Internet and energy consumption has had a high profile, but the conclusions are controversial [41].

In conclusion, the relation between the digital economy and urban green growth has a theoretical foundation established by previous research. However, there are still some deficiencies that need to be addressed. First, the current studies mainly focus on the effects of the internet or ICT (Information and Communications Technology) on economic advancement and technological innovation [42]; few scholars systematically examine the influences of the digital economy on urban green growth considering the undesirable output factors of pollution emissions. Second, there is still a need for a relatively systematic and comprehensive evaluation index system for the digital economy, a still needs to be developed. Most literature only use single indicators such as Internet development and Internet penetration to replace [43], but single indicators cannot objectively circumvent partiality. The digital economy is a relatively broad concept, and a single indicator cannot objectively represent its true level. Moreover, some research is confined to provincial-level data, and there needs to be a specialized study on the digital economy at the city level. Third, most studies focus on the overall effect, ignoring regional heterogeneity and spatial effects, which may result in biased estimates.

### 2.2. Hypotheses development

This research presents the influential mechanisms of the digital economy on urban green growth. Fig 1 illustrates our theoretical framework and hypotheses.

**Fig 1:** The theoretical framework of the digital economy on urban green growth.

#### 2.2.1. Direct effects of the digital economy on urban green growth

Green growth is an economic growth model characterized by low pollution and high efficiency [44]. Although the concept of green growth has gradually become an essential guideline for urban economic development, the economy’s green transformation still suffers from an unbalanced industrial structure, insufficient development momentum, and an imperfect development model. The digital economy, a new economic form with data as its primary factor of production [45], can significantly minimize the extensive use of physical resources in traditional industrial production, increasing the operational efficiency of resource utilization and emission reduction. Moreover, digital technology aggregates fragmented demand information with supply information by constructing a digital economy platform, reducing the search costs for enterprises and users and enhancing the efficiency of information interaction. A new generation of digital technologies is rapidly emerging as a dividend for green growth compared to traditional dividends with declining marginal effect such as land and energy [46], lowering barriers to the flow of data, technology and talent between regions. In addition, the sectors of the fast-growing digital economy are concentrated in the less ecologically harmful ICT sectors, which can cut down on energy consumption and pollution emissions by crowding out high-polluting industries [47]. A focus on the role of digital technology in fostering high-quality growth in emerging sectors may strengthen the need for digital transformation and green economy; hence, we argue:

**Hypothesis 1.** The digital economy directly drives urban green growth.

#### 2.2.2. Heterogeneous effects of the digital economy on urban green growth

Chinese cities differ in their economic advancement, resource endowments, industrial structures and technological advantages [48], indicating regional heterogeneity. Because of this, the digital economy’s contribution to urban sustainable growth will also be influenced by regional heterogeneity. Moreover, the digital divide still exists [49], making the uneven growth of the regional digital economy a matter of great concern to society. Specifically, in eastern cities, the digital economy is relatively mature and accounts for a greater share of the economy, while there are more constraints to the digital economy in the mid-western cities. Thus, it is vital to objectively examine cities’ green growth based on the attributes of regional heterogeneity. Compared with developing cities, developed cities have a comparative advantage in digital infrastructure building, application, and technology and are easier to obtain digital dividends and hence contribute more to their green growth [50]. Furthermore, changes in cities’ industrial composition might affect the regional digital economy’s growth and ecological efficiency [51]. In cities with a high concentration of industry, the technological efficiency advantages and the transformation of traditional production processes brought about by digital technology in traditional industries have the potential to unleash the pollution control and economic growth effects of the digital economy. In addition, urban agglomerations can expedite industrial reorganization and technological innovation and boost the digital economy’s dynamism; therefore, we propose:

**Hypothesis 2**
The digital economy has heterogeneous effects on urban green growth in terms of urban location, major urban agglomerations, and urban industrial structure.

#### 2.2.3. Spatial spillover effects of the digital economy on urban green growth

Compared with traditional business models, data resources and information networks are the key carriers and factors of production for the digital economy, establishing an open ecological environment and transcending the boundaries of geographical distance [52]. First, the competitive effect between neighboring regions makes inter-regional cooperation poor, and the cost of forming a well-functioning industrial agglomeration pattern is high because of spatial isolation, thereby preventing the positive externalities of industrial agglomeration and regional cooperation from being fully exploited. The digital economy makes spatial distance less of a barrier to regional economic cooperation and facilitates industrial agglomeration and information flaws across time and space between cities. Furthermore, digital tools are rapidly expanding to new sectors, accelerating the emergence of new means of resource utilization to enhance sustainable growth [53]. Second, the digital economy is the industrialization and marketization of the information technology revolution, characterized by digitization, networking and intelligence [54]. It can enhance cooperation and communication between different firms, thus improving resource use efficiency and reducing pollution emissions. Finally, digital modes can improve the transparency of environmental data to systematically disclose information about enterprises in terms of environmental governance, emissions and rewards and punishments, thereby contributing to the governance of the urban environment. Moreover, digital technology can guide transregional divisions of labor and cooperation [55], improving the efficient flow of different resource elements and controlling environmental pollution. Accordingly, the digital economy in one region can also affect the other regions’ green advancement, leading to the following hypothesis:

**Hypothesis 3.** The digital economy can affect urban green growth in neighboring regions through spatial spillover effects.

#### 2.2.4. Indirect effects of the digital economy on urban green growth

The digital economy can achieve precise matching of factors through the effects of penetration, integration, substitution, matching and universal benefit and thus promote regional green growth. The penetration effect of the digital economy is primarily reflected in the ability of digital technology to embed itself in existing factor resources and realize the digital transformation of production factors [56]. Enterprises can use information networks to search for factors online, breaking the information barrier between supply and demand of factors, effectively reducing the search cost of factors and thus alleviating resource mismatch. The digital economy has facilitated the continuous convergence of factor resources such as data and knowledge with traditional factor resources such as labor and capital, realizing complementarities and reconfigurations between factors and enhancing resource allocation efficiency [57]. Following the digital transformation of traditional factor resources, the substitution effect of the digital economy has gradually emerged. The widespread use of digital technology has promoted the substitution of capital factors for labor factors, causing simple and repetitive mechanical labor to be gradually replaced by automated production, and increasing the demand for high-end labor jobs, thus optimizing the allocation of factor resources [58]. The digital economy has also broken down the market barriers to factor resources, promoting the circulation of factor resources in a larger area and thus optimizing the combination of resources [59]. In addition, the digital economy can alleviate enterprises’ financing constraints. The widespread use of digital finance enables financial institutions to quickly screen information about enterprises, provide personalized financing services in line with their actual operating conditions, and optimize the mismatch of credit resources.

Unlike traditional economic growth, the digital economy takes on a new form, which can release the emerging dividends of green technological innovation with the development new digital technologies and fast networks [60]. Digital technologies are applied to all aspects of production and sales, increasing technological content and reducing operating costs, enabling enterprises to achieve intelligent development and operation. Moreover, the technological threshold and access costs for enterprises are significantly reduced; therefore, the cost of green technology innovation for enterprises is also significantly reduced, which has a positive promoting effect on green technology innovation [61]. The digital economy can also bring easy access to technology flows, drive high-tech talent into emerging areas of the digital economy, promote the optimization of talent resource allocation, and lay a good foundation of innovation factors for enhancing green technology innovation [62]. In addition, digital transformation can prompt enterprises to innovate their business models and compel them to enhance manufacturing technology. Meanwhile, the polluting industries are forced to shift their focus to environmental protection and sustainable innovation. Digital green technology innovation accelerates the efficient use of resources and emission reduction, minimizes the negative externalities of production and enhances the quality of green growth while fostering economic expansion; correspondingly, we argue:

**Hypothesis 4a**
The digital economy can indirectly enhance urban green growth by alleviating factor mismatch.
**Hypothesis 4b**
The digital economy can indirectly enhance urban green growth by promoting green technology innovation.

## Section 3: Data, variables, and methods

### 3.1. Data

The panel data of 279 cities in China from 2012 to 2021 are used as the samples in this research, and all original data are mainly obtained from China City Statistical Yearbook, China Information Industry Yearbook, Research Report on the Development of Chinese Government Websites, and the WIND database. Some missing data can be supplemented by interpolation or regression.

### 3.2. Variables

#### 3.2.1. Measurement of urban green growth

The explained variable is urban green growth (UGG). The measurement methods of green growth level in existing research include the target system-evaluating method and efficiency measurement method. The efficiency measurement method can be subdivided into stochastic frontier analysis (SFA) and data envelopment analysis (DEA). Compared with the SFA method, the DEA method has the advantage of evaluating multi-output or multi-input elements at the same time [63]. However, in the actual process of economic production, the inputs of labor, capital, and energy will be used to manufacture industrial goods, which will also generate pollution emissions, that is, undesirable output. The SBM model based on undesirable output can determine the relaxation of input and output and consider unexpected outputs. Thus, this model is more useful for the actual production condition and is commonly used to measure energy efficiency and ecological efficiency. Specifically, assuming there are m DMUs, and each DMU has n input, *S*_1_ expected output, and *S*_2_ unexpected output. The vector form is expressed as *x*∈*R*^*n*^, $y^{g}\in R^{S_{1}}$, $y^{b}\in R^{S_{2}}$, where *X*, *Y*^*g*^ and *Y*^*b*^ are matrices; $X=[x_{1},x_{2}\cdots x_{m}]\in R^{n\times m}$, $Y^{g}=[y_{1}^{g},y_{2}^{g}\cdots y_{n}^{g}]\in R^{S_{1}\times m}$, $Y^{b}=[y_{1}^{b},y_{2}^{b}\cdots y_{n}^{b}]\in R^{S_{2}\times m}$. *S*^−^, *S*^*g*^, and *S*^*b*^ are the slack of input, expected output, and unexpected output, respectively; *λ* is the weight vector and is used to construct the SBM-undesirable model:

$$\rho =\min\frac{1-\frac{1}{n}\sum_{i=1}^{n}\frac{s_{i}^{-}}{x_{i0}}}{1+\frac{1}{s_{1}+s_{2}}(\sum_{r=1}^{s_{1}}\frac{s_{r}^{g}}{y_{{}_{r0}}^{g}}+\sum_{r=1}^{s_{2}}\frac{s_{r}^{b}}{y_{{}_{r0}}^{b}})}$$ (1)

$$s.t.\{\begin{array}{l} x_{0}=X\lambda +S^{-}\\ y_{0}^{g}=Y^{g}\lambda -S^{g}\\ y_{0}^{b}=Y^{b}\lambda +S^{b}\\ \lambda \geq 0,S^{-}\geq 0,S^{g}\geq 0,S^{b}\geq 0 \end{array}$$ (2)

However, the SBM model still has the disadvantage of not being able to distinguish the efficiency values of the effective decision-making units (DMUs), which results in a loss of information from the effective DMUs. Tone [64] presented an unexpected output super-efficiency SBM (super-SBM) model, which combines the advantages of the super-efficiency model and the SBM model and can decompose the effective DMUs, thus avoiding the problem of information lose mentioned above. The super-SBM model is constructed as Eqs (3) and (4):

$$\rho^{*}=\min\frac{1-\frac{1}{n}\sum_{i=1}^{n}\frac{\bar{x}}{x_{i0}}}{1+\frac{1}{s_{1}+s_{2}}(\sum_{r=1}^{s_{1}}\frac{s_{r}^{g}}{y_{{}_{r0}}^{g}}+\sum_{r=1}^{s_{2}}\frac{s_{r}^{b}}{y_{{}_{r0}}^{b}})}$$ (3)

$$s.t.\{\begin{array}{l} \bar{x}\geq X\lambda \\ \bar{y^{g}}\leq Y^{g}\lambda \\ \bar{y^{b}}\geq Y^{b}\lambda \\ \bar{x}\geq x_{0},\bar{y^{g}}\leq y_{0}^{g},\bar{y^{b}}\geq y_{0}^{b},\lambda >0 \end{array}$$ (4)

where the objective function value of ρ* represents the DMUs’ efficiency values. The other variable definitions are similar to those in Eqs (1) and (2). The above models are conducted assuming constant returns to scale.

We adopt inputs, expected outputs, and unexpected outputs to calculate the green growth level. Specifically, the inputs include capital stock, labor force and resource consumption. The total fixed asset investment and fixed asset investment price index are used to measure the stock based on the “perpetual inventory method” [65]. Labor force is calculated by the total number of employees in the city. Resource consumption is represented by the area of urban building land, total water supply and total electricity consumption. The expected output is defined as urban GDP. The unexpected outputs include industrial wastewater discharge, industrial waste gas discharge, and general industrial solid waste generation. Both GDP and capital sock use 2000 constant prices.

#### 3.2.2. Measuring the digital economy level

The digital economy (DE), a relatively complex and systematic concept, is the explanatory variable in this paper. Considering that the influence of the digital economy on cities’ green growth is multi-dimensional, it is unreasonable to measure the comprehensive level of regional digital economy simply by using the industrial added value or output efficiency in the digital economy (Pan et al., 2022). Therefore, we construct a comprehensive index system reflecting the digital economy from four dimensions and apply the entropy method for calculation (see Table 1).

**Table 1:** The comprehensive index system of the digital economy.

Target level	Standard level	Index level	Indicator attribute
Digital economy	Digital industrialization	Per capita telecommunication services	+
		Number of listed companies in computer, communication and other electronic equipment manufacturing industry	+
		Number of listed companies in the software and IT services sector	+
		Proportion of information practitioners	+
	Industrial digitization	Number of listed companies in the intelligence business	+
		Number of listed companies in the e-commerce business	+
		Digital Inclusive Finance Index	+
		E-commerce market transactions	+
	Digital governance	Mobile phone penetration rate	+
		Fixed telephone penetration rate	+
		Internet broadband penetration rate	+
		China Government Website Development Index	+
	Digital sustainability	Proportion of college students	+
		Patent authorization of high-tech companies	+
		Ratio of R&D expenditure to GDP	+

#### 3.2.3. Mediating variables

Based on the previous studies, resource mismatch (RM) and green technology innovation (GTI) are selected as mediating variables to analyze the mediating effect of the digital economy on cities’ green growth level. According to the assessment method of Wu et al. [66], this study approximates the absolute distortion coefficient by calculating the relative distortion coefficient for each factor, and then obtaining the resource mismatch degree for labor (RL) and capital (RK) factors. In addition, green technology innovation, one of the important influencing factors for promoting green growth (Wang et al., 2021), can be represented by the ratio of the number of authorized green patents to total green patent applications at the city level, which can exclude other unobservable factors and represent actual green innovation capacity.

#### 3.2.4. Control variables

After referring to the relevant literature [67], this paper selects 5 indicators that may affect urban green growth as control variables: (1) Economic development level (ECO). A region with a higher level of economic development has better endowment conditions, which not only provide sufficient capital for the transformation and upgrading of the city, but also help attract resources and talents to gather and have the foundation for the realization of green growth. The logarithm of cities’ per capita GDP is used for this measure. (2) Foreign direct investment (FDI). The inflow of foreign capital will be accompanied by the introduction of advanced production technologies and environmentally friendly business concepts, promoting the transformation of local development models. However, foreign investment may cause the transfer of backward production capacity from abroad to the region, exacerbating local environmental pollution. The ratio of actual foreign capital use to GDP represents foreign direct investment. (3) Industrial structure (IND). Currently, China has a high proportion of traditional industries with high energy consumption, high emissions and low efficiency. The high proportion of industry in the industrial structure of a city will hinder its industry’s green transformation. The ratio of the added value of the secondary sector to GDP measures industrial structure. (4) Urbanization (URB). A city with a higher level of urbanization has more significant advantages in terms of industrial structure, population quality, management mechanisms and development concepts, thus contributing to local green growth. Urbanization is represented by the proportion of urban resident population to the total population. (5) Environmental regulation (ER). Increased regional environmental regulation can increase the pollution cost of enterprises and promote their autonomous transformation and upgrading in the region, thereby achieving regional green growth. We adopt the comprehensive utilization rate of municipal general solid waste to measure urban environmental regulation. The descriptive statistics of the variables are presented in Table 2.

**Table 2:** Descriptive statistics.

Variables	Obs.	Mean	Std. Dev.	Min	Max
UGG	2790	0.6257	0.2164	0.0185	1.0000
DE	2790	1.6977	0.7708	1.1520	6.6322
GTI	2790	0.4417	0.2478	0.0065	0.8825
RL	2790	0.5532	0.4023	0.0048	2.5547
RK	2790	0.2427	0.1031	0.0101	0.9138
ECO	2790	1.9257	1.1142	0.0876	12.1548
FDI	2790	0.3226	0.3576	0.0094	1.9041
IND	2790	0.3034	0.0230	0.0249	0.5434
URB	2790	0.6147	0.3929	0.3223	0.9981
ER	2790	0.4616	0.3684	0.1329	1.0000

### 3.3. Econometric methods

This paper presents a benchmark model for investigating the relationship between the digital economy and urban green growth. The specific mathematical expression is as follows:

$$UGG_{it}=\alpha_{0}+\alpha_{1}DE_{it}+\alpha_{2}Controls_{it}+\mu_{i}+\delta_{t}+\varepsilon_{it}$$ (5)

where i and t represent city and time; *UGG*_*it*_ is green growth level; *DE*_*it*_ is the digital economy; *Controls*_*it*_ means the control variables; *μ*_*i*_ denotes the individual fixed effect and *δ*_*t*_ denotes the time-fixed effect; *ε*_*it*_ refers to the random disturbance term.

This study also assesses whether green technology innovation and resource mismatch have potential indirect effects in the mechanisms. Based on the stepwise regression method, the mediating effect model is constructed and shown in Eqs (6) and (7).

$$Med_{it}=\theta_{0}+\theta_{1}DE_{it}+\theta_{2}Controls_{it}+\mu_{i}+\delta_{t}+\varepsilon_{it}$$ (6)

$$UGG_{it}=\phi_{0}+\phi_{1}Med_{it}+\phi_{2}DE_{it}+\phi_{3}Controls_{it}+\mu_{i}+\delta_{t}+\varepsilon_{it}$$ (7)

where *Med*_*it*_ represents the mediating variables, including green technology innovation and resource mismatch. Eq (5), Eq (6) and Eq (7) together constitute the mediating effect model. Eq (5) evaluates the impact of the digital economy on urban green growth; Eq (6) evaluates the effects of the digital economy on mediating variables, and Eq (7) evaluates the effects of the digital economy and the mediating variables on urban green growth. When *α*_1_ in Eq (5) is significant, it means that the digital economy has a significant impact on urban green growth, and then, we test whether *θ*_1_ in Eq (6) and *ϕ*_1_ in Eq (7) are significant. If *θ*_1_ and *ϕ*_1_ are both significant, it suggests that the digital economy can affect urban green growth through the mediating variables. Meanwhile, if *ϕ*_2_ is also significant, it indicates that the digital economy directly affects urban green growth through the influence of the mediating variables.

The theoretical analysis and existing studies have proved that the digital economy affects urban green growth in the local region and has a strong spatial correlation with urban green growth in the surrounding regions. It will lead to biased estimation results if the empirical study of this article neglects the existence of spatial spillover effects. Consequently, Eq (5) is extended spatially by incorporating the spatial term of the digital economy and urban green growth in the model to control its spatial correlation. Traditional OLS estimates can only evaluate the effects of the digital economy on urban green growth from the perspective of intra-city. The spatial Durbin model (SDM) will reflect the spatial correlation caused by explanatory variables or explained variables or error terms [68]. It can still obtain unbiased regression coefficients even if the spatial lag model (SLM) or spatial error model (SEM) should be adopted for real data [69]. The spatial Durbin model in this paper is constructed as follows:

$$\begin{array}{l} UGG_{it}=\beta_{0}+\rho \sum_{j=1}^{n}W_{ij}UGG_{jt}+\beta_{1}DE_{it}+\beta_{2}\sum_{j=1}^{n}W_{ij}DE_{jt}\\ \;+\beta_{3}Controls_{it}+\beta_{4}\sum_{j=1}^{n}W_{ij}Controls_{jt}+\mu_{i}+\delta_{t}+\varepsilon_{it} \end{array}$$ (8)

where *ρ* denotes the spatial spillover coefficient of urban green growth; *β*_0_, *β*_1_, *β*_2_, *β*_3_, and *β*_4_ are the coefficients; *W*_*ij*_ indicates an *N*×*N* order spatial weight matrix. The adjacent spatial weight matrix and geographic distance spatial weight matrix are selected in this article. The Equation of the adjacent spatial weight matrix can be defined as follows:

$$W_{ij}^{a}=\{\begin{array}{l} 1,\;i\neq j\\ 0,\;i=j \end{array}$$ (9)

where city i has a common boundary with city j; then, *W*_*it*_ = 1; otherwise, *W*_*it*_ = 0.

The geographic distance spatial weight matrix can be defined as follows:

$$W_{ij}{}^{g}=\{\begin{array}{l} \frac{1}{d_{ij}^{2}},\;i\neq j\\ 0,\;i=j \end{array}$$ (10)

where *d*_*ij*_ denotes the surface distance between cities calculated by the location information (longitude and latitude).

## Section 4: Empirical results and discussion

### 4.1. Baseline results

We investigate the influence of the digital economy on urban green growth using model (5). The benchmark regression results are detailed in Table 3. As is demonstrated in Column (1), when only individual and time fixed effects are controlled, the estimated coefficient of the digital economy is significantly positive at the significance level of 1%. Furthermore, after gradually adding the control variables, the digital economy’s coefficient is still positive and significant. These findings suggest that the digital economy can drive urban green growth. From the results in Column (6), which contains all the control variables, we can infer that each unit increase in the digital economy has a positive effect on cities’ green growth level by 0.0563 percentage points. The similar results are obtained by Wei [24]. The results of the baseline regression model validate Hypothesis 1, which indicates that the higher the level of the digital economy, the higher the level of cities’ green growth.

**Table 3:** Baseline findings.

Variables	UGG (1)	UGG (2)	UGG (3)	UGG (4)	UGG (5)	UGG (6)
DE	0.0241*** (3.11)	0.0465*** (3.63)	0.0496*** (3.83)	0.0507*** (4.58)	0.0558*** (5.07)	0.0563*** (6.10)
ECO		0.0701*** (4.82)	0.0646*** (4.27)	0.0610*** (3.58)	0.0621*** (4.15)	0.0671*** (4.40)
FDI			-0.0111 (-1.46)	-0.0098 (-1.20)	-0.0103 (-1.38)	-0.0086 (-1.06)
IND				-0.0220*** (-2.68)	-0.0151** (-2.26)	-0.0115** (-2.12)
URB					0.00146** (2.15)	0.0094* (1.85)
ER						0.0105** (2.13)
Constant	0.5330*** (5.04)	0.5212*** (4.69)	0.4039*** (6.22)	0.5595*** (7.37)	0.6682*** (8.05)	0.7371*** (8.89)
City FE	YES	YES	YES	YES	YES	YES
Year FE	YES	YES	YES	YES	YES	YES
Observations	2790	2790	2790	2790	2790	2790
R-squared	0.1419	0.1609	0.1671	0.1734	0.1772	0.1784

Note

*p < 0.1

** p < 0.05

*** p < 0.01. T-statistics are in parentheses. (the same below)

Moreover, the results of Column (6), including all the control variables, demonstrate that the economic development level (ECO) has positive effects on cities’ green growth, showing that the higher the level of urban economic development, the more conducive to achieving green growth. With a negative coefficient, foreign direct investment (FDI) fails to pass the significance test. A possible explanation is that most cities introduce low-level foreign capital, creating industrial pollution and hampering local green growth. This finding confirms the “Pollution Refuge Hypothesis”, highlighting the significance of high-quality FDI in fostering a city’s green and sustainable development. Industrial structure (IND) is significantly negative at the 5% level, revealing that the industrial structure with a high proportion of industry can suppress cities’ green growth. Urbanization (URB) positively affects urban green growth, illustrating that urbanization promotes cities’ green growth. The primary reason for this phenomenon is that improving urbanization level can enhance the concentration of resources and the overall operation quality and promote the efficiency of urban green growth. Environmental regulation (ER) positively leads to an increase in urban green growth, revealing that cities’ strong environmental protection can boost green growth.

### 4.2. Robustness check

Some robustness checks were performed to establish the reliability of the findings of the benchmark regression model. First, the COVID-19 pandemic poses a substantial risk to our lives and hinders China’s economic progress. To eliminate the effects of the COVID-19 pandemic in 2020, we exclude the sample data for 2020 in the regression analysis. Moreover, China’s municipalities are significantly higher than ordinary prefecture-level cities in terms of economy, population and area. Thus, the development of their digital economy may differ significantly from that of prefecture-level cities. We further excluded the sample data from Beijing, Shanghai, Tianjin and Chongqing for testing. the coefficients of all control variables will no longer be provided for the purpose of brevity. Columns (1) and (2) of Table 4 show the findings for the sample subinterval estimates. The estimated coefficients of the digital economy remain significantly positive, demonstrating that the positive relation between the digital economy and urban green growth is robust even when excluding special samples.

**Table 4:** Robustness check.

Variables	UGG (1)	UGG (2)	UGG (3)	UGG (4)	UGG (5)	UGG (6)
DE	0.0519*** (5.44)	0.0491*** (5.03)	0.0630*** (6.26)			0.0531*** (5.86)
DE(t-1)				0.0617*** (6.12)		
DE(t-2)					0.0693*** (7.59)	
Constant	0.9540*** (8.19)	0.8422*** (5.28)	0.9221*** (6.15)	0.9163*** (7.33)	0.7767*** (5.73)	0.0808*** (6.51)
Controls	YES	YES	YES	YES	YES	YES
City FE	YES	YES	YES	YES	YES	YES
Year FE	YES	YES	YES	YES	YES	YES
Observations	2511	2750	2790	2511	2232	2790
R-squared	0.1705	0.1689	0.1853	0.1732	0.1865	0.1731
Kleibergen-Paap rk LM statistic						575.387 [0.0000]
Kleibergen-Paap rk Wald F statistic						461.975 {95.56}
F-statistic						6.2645

Note: P-value in square brackets. The critical value at the 10% level of weak identification test in brace.

Second, two control variables (financial development (FIN) and education level (EDU)) are added to the benchmark model to solve the endogeneity problem brought on by missing variables. Specifically, financial development is measured by the ratio of the balance of deposits and loans of financial institutions to GDP, and education is represented by the number of students enrolled in high education institutions. The regression findings are shown in Column (3). The digital economy’s regression coefficient is positive and significant, revealing that the digital economy still significantly promotes a city’s green growth.

Third, cities with a high level of green growth are inclined to create digital technologies, hence fostering a higher level of the digital economy. To deal with this endogeneity, we select the digital economy data by lagging 1 and 2 for the benchmark model. In Columns (4) and (5), the digital economy’ coefficients are significantly positive in two cases, demonstrating a positive relationship between the digital economy and urban green growth. In the lagged model, the digital economy’s coefficients are increasing, indicating that the driving role of the digital economy to cities’ green growth is expanding with the increase of the lag order, and the long-term impact of the digital economy is greater compared with the short-term impact.

Fourth, an instrumental variable method can better alleviate the potential endogeneity. By referring to Nunn and Qian [70], we create the interaction term (HDel) as an appropriate instrumental variable using the number of post and telecommunications bureaus per million in 1984 and China’s internet users in the past year. The two stage least square method is used for estimation. The results in Column (6) of Table 4 again confirm that the digital economy has a significant contribution to cities’ green growth after adopting the instrumental variable. The Kleibergen-Paap rk LM statistic and the Kleibergen-Paap rk Wald F-statistic reject the null hypothesis, demonstrating it has passed the endogenous test. Thus, the above findings are highly consistent with the benchmark regression results, providing more evidence that the core conclusion is robust.

### 4.3. Heterogeneous analysis

To examine the heterogeneous impact of the digital economy on urban green growth, we perform a subsample regression based on prior hypotheses on the effect of the digital economy on urban green growth from three characteristics of urban location, major urban agglomerations, and urban industrial structure. We divide the urban location category into groups according to standard of cities in the eastern region and mid-western regions of China, including the Yangtze river delta, Beijing-Tianjing-Hebei delta, and the Pearl river delta as the key urban agglomeration samples; others are classified as non-key. Furthermore, the advanced industrial structure is measured by the ratio of the value-added of the tertiary industry to the value-added of the secondary industry. Thus, cities with an industrial structure level above national average are considered as high-level cities, while others are deemed low-level cities.

Table 5 shows the findings of heterogeneity testing. The results reveal that the digital economy exerts positive effects on green growth in eastern cities, major urban agglomerations, and high-level cities, but has little impact on that in other cities. Hypothesis 2 is verified. A possible explanation for this finding is that the digital dividends are fully released to better foster green growth in eastern cities, major urban agglomerations, and high-level cities. These cities have developed infrastructure and advanced digital technologies; thus, developing the digital economy can harness these first-mover advantages to strengthen social and economic systems and promote regional economic advancement in terms of quality and efficiency. Conversely, the digital economy is still in its infancy and has yet to form a scale effect in mid-western cities, non-major urban agglomerations, and low-level cities. This shows the green effect of the digital economy is not evident in these cities.

**Table 5:** Heterogeneity analysis.

Variables	Eastern	Mid-western	Major	Non-major	High-level	Low-level
	UGG (1)	UGG (2)	UGG (3)	UGG (4)	UGG (5)	UGG (6)
DT	0.0566*** (5.73)	0.0453 (1.19)	0.0538*** (3.52)	0.0411 (1.08)	0.0515** (2.35)	0.0470 (1.39)
Constant	0.7338*** (8.43)	0.7762*** (8.79)	0.6589*** (7.12)	0.5765*** (6.27)	0.6161*** (6.81)	0.5360*** (5.45)
Controls	YES	YES	YES	YES	YES	YES
City FE	YES	YES	YES	YES	YES	YES
Year FE	YES	YES	YES	YES	YES	YES
Observations	1020	1770	810	1980	1140	1650
R-squared	0.1673	0.1697	0.1538	0.1505	0.1611	0.1429

### 4.4. Spatial spillover effects

Moran’s I method is used to test the spatial correlation of the core variables before spatial econometric analysis. Table 6 demonstrates the findings of the spatial correlation test. The Moran’s index values for the digital economy and urban green growth under the adjacent weight matrix and geographic weight matrix are mostly positive and significant, and the null hypothesis of no spatial correlation is significantly rejected, revealing that the spatial spillover effects can be further examined in this research.

**Table 6:** The spatial correlation test.

Year	*W* ^*a*^	*W* ^*g*^	*W* ^*a*^	*W* ^*g*^
	DE (1)	DE (2)	UGG (3)	UGG (4)
2012	0.065***	0.258***	0.036***	0.049***
2013	0.061***	0.259***	0.030***	0.042***
2014	0.062***	0.255***	0.025***	0.013
2015	0.041***	0.239***	0.027***	0.035**
2016	0.065***	0.260***	0.019**	0.054***
2017	0.076***	0.267***	0.018***	0.062***
2018	0.060***	0.260***	0.019**	0.021*
2019	0.070***	0.267***	0.010*	0.014***
2020	0.058***	0.258***	0.020***	0.023*
2021	0.059***	0.218***	0.016**	0.051***

Table 7 presents the spatial effect regression findings under the two weight matrixes. The digital economy’s coefficients are significantly positive and pass the significance test of 1% or 5%, which are basically consistent with the results of the benchmark model, indicating the robustness of the core conclusion in this research. Furthermore, the spatial correlation coefficients *ρ* in the SDM model are significantly positive and pass the significance test of 1%, demonstrating that the digital economy has a significant spatial spillover effect. Given that point estimation testing of spatial spillover effects may result in estimation bias, it is required to decompose the overall effect into direct effect and indirect effect to precisely describe spatial spillover effects [71]. Table 7 reveals that the direct effect, indirect effect, and total effect of the digital economy on urban green growth under different weight matrix are all significantly positive. This indicates that the digital economy can effectively accelerate local green growth, and enhance neighboring cities’ green growth through spatial spillover effects, which confirms Hypothesis 3.

**Table 7:** Spatial effect estimation results.

Variables	*W* ^*a*^	*W* ^*g*^	*W* ^*a*^	*W* ^*g*^
	UGG (1)	UGG (2)	UGG (3)	UGG (4)
DE	0.0738*** (6.16)	0.0435*** (3.67)	0.0506*** (4.74)	0.0386** (2.35)
spatial rho	0.0358*** (5.34)	0.0329*** (5.12)	0.0292*** (4.19)	0.0269** (2.16)
Direct effect	0.0680*** (5.64)	0.0362*** (3.38)	0.0426*** (3.39)	0.0317** (2.36)
Indirect effect	0.0241** (2.16)	0.0224* (1.87)	0.0212** (3.32)	0.0193** (2.18)
Total effect	0.0921** (2.39)	0.0586** (2.07)	0.0638*** (2.37)	0.0510*** (3.51)
Controls	NO	NO	YES	YES
City FE	YES	YES	YES	YES
Year FE	YES	YES	YES	YES
Observations	2790	2790	2790	2790
R-squared	0.1482	0.1415	0.1605	0.1583
Log-pseudolikehood	264.0301	256.3271	269.4239	267.9231

### 4.5. Mediating effects

Table 8 shows the estimation findings of the mediating effects. Columns (1) and (3) reveal that the regression coefficients of the digital economy on labor resource mismatch and capital resource mismatch are both significantly negative (-0.0614 and -0.4835), suggesting that the digital economy can reduce urban resource mismatch. As shown in Columns (2) and (4), the estimated coefficients for the relation between labor resource mismatch and capital resource mismatch and urban green growth are also significantly negative (-0.2085 and -0.0283), but the regression coefficients of the digital economy have decreased, indicating that the digital economy can indirectly drive the urban green growth level by reducing the resource mismatch of labor and capital. Moreover, we can obtain the indirect effects of the digital economy on urban green growth are 0.0128 (-0.0614×-0.2085 = 0.0128) and 0.0137 (-0.4835×-0.0283 = 0.0137), respectively. Hypothesis 4a is verified. The digital economy’s development can accelerate the reorganization of cross-regional funds, technology and other production factors and effectively integrate the cross-regional resource elements, thereby reducing resource mismatch and improving urban green growth.

**Table 8:** Mediating effects.

Variables	RL (1)	UGG (2)	RK (3)	UGG (4)	GMI (5)	UGG (6)
DE	-0.0614*** (-5.44)	0.0435*** (4.46)	-0.4835*** (-13.26)	0.0426*** (4.27)	0.2362*** (11.94)	0.0517*** (5.72)
GMI		-0.2085*** (-8.35)				
RL				-0.0283*** (-3.11)		
RK						0.0195*** (2.89)
Constant	1.7472*** (18.61)	1.8166*** (19.28)	1.5667*** (17.74)	2.0213*** (23.74)	1.3905*** (15.14)	1.4445*** (16.59)
Controls	YES	YES	YES	YES	YES	YES
City FE	YES	YES	YES	YES	YES	YES
Year FE	YES	YES	YES	YES	YES	YES
Observations	2511	2750	2790	2511	2232	2790
R-squared	0.2529	0.3961	0.2946	0.3629	0.3541	0.4148

The impact of the digital economy on green technology innovation is significantly positive in Column (5), demonstrating that it can enhance green technology innovation. The effect of the digital economy on urban green growth is also significantly positive, but the digital economy’s estimated coefficient has decreased from 0.0563 to 0.0517, indicating that the digital economy can indirectly drive urban green growth through the positive mediating effect of cities’ green technology innovation. The indirect effect is 0.0046 (0.2362×0.0195 = 0.0046). Hypothesis 4b is confirmed. The digital economy, with digital technology as the core driving force, can improve the utilization of energy technology, lowering pollution emissions in firms, and exerting positive effects on urban green growth.

## Section 5: Conclusions and policy implications

From a multidimensional perspective, this research uses Chinese urban panel data to investigate the influence mechanisms of the digital economy on urban green growth. The findings show that the digital economy can effectively promote cities’ green growth. Furthermore, there is a significant heterogeneity effect across cities, with the release of digital dividends being more efficient in the eastern cities, major urban agglomerations, and high-level cities. Additionally, the digital economy can improve both local green growth and the green growth of the neighboring cities through spatial spillover effects. We further investigate the transmission mechanisms, and confirm that the digital economy can indirectly drive urban green growth by reducing resource mismatch and enhancing green technology innovation.

Some worthy policy implications emerge from the above empirical analysis results. First, the government should further raise investment in the infrastructures essential for the digital economy, such as promoting the construction of new infrastructure including artificial intelligence, cloud platform and 5G. Different cities need to maximize the role of digital technologies in facilitating China’s economic restructuring and enhance the deep integration of traditional industries with digital technologies. This can improve the resource utilization efficiency of traditional industries and reduce production costs and pollution emissions, realizing traditional industries’ digital and green growth. Second, a huge digital divide between cities still exists, which can weaken the spillover effects of the digital economy on urban green growth. The superior government should assist less developed regions catch up through institution and policy benefits. Local governments should strengthen inter-regional cooperation to form an advantageous ecology of mutual integration and promotion, thus driving cities’ digital transformation and green innovation. Third, the government needs to make use of digital technologies to optimize the allocation of resources, thereby actively enhancing the role of the digital economy in reducing resource mismatch. Moreover, it is necessary for the government to further promote the widespread use of digital technologies to achieve effective integration of innovation factors such as funds, talent and technology. This strategy is conducive to enhancing enterprises’ production technology, energy-saving technology and environmental protection technology, thus facilitating the transformation and upgrading of traditional industries and promoting green growth.

This research provides a preliminary discussion about the role of the digital economy in urban green growth, but much remains to be done. First, this article uses a combination of theoretical hypotheses and empirical tests to undertake the relevant research, which may be extended and analyzed from different perspectives. Future studies could seek to establish a theoretical model for exploring the relation between the digital economy and urban green growth. Second, although the research investigates many Chinese cities, we could not analyze data from all Chinese cities due to data unavailability. In addition, as we have only explored the mechanisms of resource mismatch and green technology innovation on urban green growth, future research should examine other possible mechanisms, such as environmental regulation and digital governance. Finally, using China as an example may restrict the results’ generalizability. This model might be used to investigate how the digital economy affects urban green growth in other emerging countries.
